# The Management of Educational Talents in Vocational Colleges Based on Wireless Network in the Artificial Intelligence Era

This article has been retracted.

**DOI:** 10.1155/2022/2298139

**Published:** 2022-06-24

**Authors:** Yang Zhang, Ce Wang

**Affiliations:** ^1^College of Modern Service, Harbin Vocational College of Science and Technology, Harbin 150300, China; ^2^College of General Education, Heilongjiang Polytechnic, Harbin 150080, China

## Abstract

Faced with the AI (artificial intelligence) era, it is both theoretically and practically important to examine the challenges and opportunities that vocational college education in China faces, as well as to actively explore how vocational college education can overcome the challenges and achieve a realistic path. This paper proposes and implements a wireless network-based vocational college talent management system. The main personnel management system primarily completes business operations related to daily personnel file management, while the data mining subsystem mines talent data using the DT (decision tree) classification algorithm to aid talent selection. At the same time, a new topology optimization algorithm based on the principle of minimum rigidity graph is proposed for talent management system wireless network optimization. The maximum-minimum balance criterion and the user-by-user optimization mechanism are designed to obtain the optimal relay selection and subchannel allocation strategy, ensuring the system's reliability and fairness. The optimized algorithm has a user security satisfaction of 0.93 in the range of 250 m, which is higher than other algorithms. It demonstrates that this algorithm's communication link is short, and it has good network connectivity and structural stability.

## 1. Introduction

The essence of the reform of vocational talents training education mode is to change the types of talents to meet the needs of different types of talents in different periods and societies. Talent training mode mainly includes training objectives, training norms, training methods, and finally what kind of people to train. In recent years, Internet giants have devoted themselves to the research and development of driverless technology, constantly exploring and innovating, realizing the integration of AI (artificial intelligence) [1] and traditional automobile technology, which has triggered people's endless reverie of future intelligence. From the perspective of the AI era, people gradually realize that innovative engineering and technical talents are more in line with the needs of this social and industrial transformation.

Only by deeply studying the basic theory of vocational college education can we formulate scientific policies and guidelines to guide the development of vocational college education. As the standard and requirement of training talents in schools at all levels, the goal of training talents is of great significance to the whole education and the development of specific majors in specific schools. Stukalina pointed out that the typical application of AI in education mainly includes intelligent tutors assisting individualized teaching and learning [2]. Ginsburg et al. studied AI as a course and pointed out that it is of great significance to carry out AI education courses in vocational colleges [3]. Leńko-Szymańska suggested that AI should also play a role in motor skill learning [4]. He pointed out that many learning tasks need to be completed through repeated movements, such as learning to write, draw, play musical instruments, practice motor skills, dance, and use sign language. Derosa et al. believe that “standardized work” is easily replaced by AI, while creative work and those with “emotional color and artistic creation” are difficult to replace, resulting in the phenomenon of “intermediate skills being squeezed” [5]. Filho et al. think that we should improve the combination of production and learning, combine “decentralized teaching” to innovate the classroom, and construct an effective interdisciplinary compound model [6].

AI is essentially a technological revolution. When artificial intelligence (AI) continues to profoundly influence and change human production and life, vocational college education, as one of the factors of production, will inevitably be forced to actively consider how to deal with AI's arrival [7, 8]. Although AI is not human intelligence, technology products that contain AI act as a “carrier” for human intelligence, allowing them to think like humans and even surpassing human intelligence. This paper discusses the causes of some problems that exist in the innovation and development of engineering and technical talents in reality and offers suggestions for cultivating innovative talents, based on the fact that a new generation AI technology has entered the application stage. The following two aspects of this paper's innovation: (1) this paper constructs a vocational college education talent management system with a wireless network by studying the application of DT technology in talent management and using wireless network technology, with the goal of assisting enterprises in making talent management decisions and (2) the topology optimization algorithm is used to design and optimize the system database objects during the development process. It increases the readability of system design documents and provides a solid foundation for the system's implementation.

## 2. Related Work

### 2.1. Talent Management Research

With the continuous development of science and technology, mankind has gradually entered the era of the knowledge economy. In the era of the knowledge economy, it means that the development and renewal of knowledge become more and more valuable. As an important factor of production in people's lives, it has been widely accepted by people. The goal of talent cultivation plays a very important role in the whole vocational college education system. It is not only the starting point of practical education activities but also the standard to evaluate the success of a school. Judging from the orientation of talent training objectives, talent training objectives can be divided into national, higher vocational, and professional training objectives.

Zheng et al., from the perspective of AI's development's demand for social talents and its impact on the employment of vocational college graduates, discussed how vocational colleges should innovate the talent training mode to promote the talent training of vocational college education to adapt to the new market demand as soon as possible [9]. Sun et al. defined the training goal of higher vocational talents as training knowledge-based skilled talents, who have both a high level of professional theoretical knowledge and a high level of operational skills [10]. Chen analyzed the factors influencing the change of talent training objectives from five aspects, namely [11], the change of social and economic development mode, the transformation and upgrading of industry and the changes and requirements of market demand, the basic law of higher vocational colleges' education, the value pursuit of higher vocational colleges' education, and the change of social talent view. Dong et al. put forward the strategies to improve the training objectives of educational talents in higher vocational colleges under the reform of the education supply side: strengthening specialty construction, strengthening the integration of production and education and school-enterprise integration and reforming the school-running mode [12]. Yang said that if education cannot make the workforce acquire new skills in time, the mismatch between the skills required by new technologies and those provided by the workforce will hinder the transformation [13]. Wei and others think that both teaching and practice should be devoted to innovation [14]. Jian believes that compound talents should be cultivated in the AI era [15].

### 2.2. Research on Wireless Network Optimization

Wireless network optimization is a series of processes to obtain relatively stable network coverage, capacity, and quality through certain economic investment so as to obtain better performance. For wireless sensor networks with limited power, topology optimization can reduce power consumption, prolong the life cycle of the network, improve the stability of communication link structure, and make the network better used in a complex environment.

Sagduyu et al. proposed a four-level clustering algorithm, which considered the problem of residual energy between nodes, built a hierarchical link structure, and improved the network load balance [16]. However, when more clusters are generated, the node degree of the head node will increase rapidly, which will affect the connectivity of the sensor. Xiao et al. proposed a robust control algorithm, which introduced the node scheduling adjustment factor and quantified the network node degree, sought the value rule of the node degree, obtained the optimal node degree of the network, and improved the balance of the network structure [17]. A method of network positioning based on stiffness matrix characteristics of the rigid graph is proposed. In the positioning process, the selection of positioning points and the construction of the network improve the eigenvalue of the stiffness matrix of the generated network, which improves the stability of the network structure on the premise of ensuring network connectivity. However, the influence of link weights on network lifetime is not considered in the algorithm.

Zhang et al. proposed a joint power tying and subchannel allocation algorithm, which can improve the capacity of the Femtocell network and protect the communication service quality of macrocell users [18]. Wang et al. have done relevant research on soft frequency reuse technology in home base station network [19]. This technology has improved the degree of reuse. Based on Wang's noncooperative game theory, the energy efficiency of a mobile communication network is maximized by appropriate power control strategies [20]. Singh et al. proposed a noncooperative game power control algorithm to optimize the network energy efficiency. In order to reduce the complexity, the author adopted distributed solution, which effectively reduced the algorithm complexity while improving the network energy efficiency [21]. Daniel et al. put forward an energy-saving subchannel allocation strategy, but this strategy does not consider the interference to neighboring cells and is not suitable for multicell scenarios, which has certain limitations [22]. Kakadia et al. put forward a medium-sized node selection strategy based on the principle of minimum outage probability, which improves the total capacity of the system and reduces the outage probability by selecting the relay with the minimum outage probability from end to end for forwarding service [23].

## 3. Methodology

### 3.1. Design of Educational Talent Management System in Vocational Colleges Based on Wireless Network

Workers in the AI era will most likely be product designers, producers, or sellers. Workers will learn how to not only understand technology but also how to maintain and debug products, as well as how to communicate with various customers to meet their needs. Many traditional industries are disappearing in the AI era, with the rapid development of science and technology, as well as the continuous application of industrial robots, while many new industries emerge. To adapt to changes in industry structure, vocational colleges should actively adjust their career scenes in response to changes in market talent supply and demand. The traditional management system falls short of meeting the modern talent management business needs. The new system, which is based on the old system, absorbs new user requirements and can meet those requirements in the workplace. As a result, the system's feasibility is strong, and it is critical to improve user satisfaction and employee productivity.

The requirement to adapt to the transformation of business forms in the AI era is to discover new technologies with creativity. Engineering and technical professionals with advanced technologies and a knack for technological innovation are unquestionably in demand. Only engineers with such abilities will be able to stand out in a sea of technological change and gain the first opportunity for personal growth. New tools, new applications, new methods, and so on will continue to emerge as new technologies inspire and support them. Engineers must make efforts in all aspects, whether in the chemical and pharmaceutical industry or in the construction and processing industry. Only in this manner can technical capability and business level meet real-world requirements. The SaaS (software-as-a-service) model is a new software application model that is gradually emerging against the backdrop of the continued maturation of application software and the in-depth development of Internet technology.

The SaaS model has the following advantages:

1. Each unit does not need to be equipped with special professional technicians to maintain the system. At the same time, access to the latest technology applications to meet changing needs;
2. There is no need for each unit to build its own management platform, and there is no need to consider issues such as cost depreciation and subsequent platform upgrade, which can effectively alleviate the pressure of insufficient funds.

In a word, building a talent management system using SaaS model can greatly reduce the burden of building and maintaining infrastructure and applications in each unit. All units can rely on the unified management platform of provinces, cities, and counties to use management software conveniently, without a large amount of hardware and software investment.

According to the concept of the SaaS model, the author initially constructed a talent management platform, and its architecture is shown in Figure 1:

The framework layer is responsible for data transmission and monitoring of the application service layer and the application integration layer, including security services, application monitoring, data backup, network control, operation management, and so on. It is the basic running environment of SaaS. The model provides application services provided by many software vendors, which ensures the high reliability, high security, and high scalability of the whole system. According to the needs for talent training in the AI era, the main modules of the designed system include talent information continuous maintenance module, business declaration module, declaration confirmation and audit module, talent and employee file management module, SMS sending and receiving module, system background management module, and so on. The system module structure is shown in Figure 2.

Compiling talent information maintenance is one of them, and it consists of two submodules: talent information registration and talent information editing. Professional title declaration and talent development special fund declaration are two submodules of the business declaration module. Two small modules are included in the application and audit module: professional title application and special fund for talent development application and audit. Six small modules make up the talent and personnel file management module: talent file transfer application, transfer application approval, file information record, transfer application file, transfer application approval, and file transfer.

DT (decision tree) module will automatically complete the whole data extraction process, and users can use the provided parameters to adjust DT so that the prediction results are more ideal. These parameters include confidence pruning and whether to merge discrete attributes. Pruning confidence determines the severity of the pruning operation and is the most important parameter. If the user makes a prediction according to the rule set when making a prediction, in the prediction module, the rule set is read from the rule file, and then its prediction data is read. In the process of prediction, a test case may predict different classification results according to different rules, and these results may contradict each other.

Considering the strong independence of this module, in order to reduce duplication of work, the system is changed to a web system, the codes of the DT generation module and prediction module are packaged in a DLL file independently, and the mining part is completed by calling dynamic link library system. In the stage of system design, DT module code design is the key and difficult point. As an independent subsystem of the talent management system, the data mining subsystem is mainly used by business decision-makers to support business talent management decisions. It includes three parts: the decision of outstanding talents, the decision of employee loyalty, and the decision of employee employment. Its structure is shown in Figure 3.

The model mainly selects the specific attributes according to the related contents of the talent index system established by the human resource management model. The indexes that reflect talent include education index, professional title index, age index, and industry index, and their credibility is proved by statistical methods.

According to business analysis, the conceptual database schema's common entity model structure, multivalued attributes, and entity relationships are transformed into a relational schema, which is then standardized. Every nonprimary attribute is functionally dependent on the relational schema code; the relationship ensures that each attribute's value range is a simple and indivisible data element. During the development process, staff not only can use out-of-the-box programme functions to operate the process but also can create many flexible processing links in the programme, and some functions and operation modules can be added, modified, and manually modified. This creates a good flexible space for system users, transforming the rigid programme into a living programme, and allowing them to experience the system's flexibility and humanized design ideas.

### 3.2. Wireless Network Optimization of Talent Management System

The era of AI is the era of machine revolution, and human-machine interaction is becoming more widespread. Many production processes necessitate the involvement of AI teams. Faced with the development situation in which start-up companies require a large number of AI talents, the talents trained by vocational colleges' original talent training objectives can no longer fully meet the new labor market demands. As a result, talent training objectives must be reset, and a new talent training plan must be developed, with the goal of meeting the new labor market demand for talents in the AI era and balancing the supply and demand of talents at the training end. All database access tasks are built in the database access class to improve the efficiency of project development and the speed of system execution. As a result, the database's public class is created and saved in the public class folder. The database control class can be called from the global module. A global file is configured in addition to the public class for accessing the database, in which the user name and password for accessing the database are stored in ciphertext form. This design method is adaptable and has a high rate of code reuse.

This paper presents a topology control algorithm for wireless sensor networks based on the optimization of algebraic stiffness characteristics of a minimum rigid body graph. The algorithm comprehensively considers the weight of communication links in the generated topological link graph and the rigidity of the generated rigid graph, which not only ensures the short communication links but also helps prolong the life cycle of the network, making the generated communication link graph more efficient and more stable in structure. The attenuation factor model is mainly used to predict the propagation loss in buildings and can deal with the influence of building types and the changes caused by obstacles. The model is flexible, and the standard deviation between the expected results and the measured values is small, while the deviation from the logarithmic distance model is much smaller. The attenuation model is

(1) $$\begin{array}{c} \bar{L}\left(d\right)=\bar{L}\left(d_{0}\right)+10\gamma_{SE}\log_{10}\left(\frac{d}{d_{0}}\right)+ad+FAF, \end{array}$$

where *d*_0_ represents the standard reference distance, taking the empirical value of 1 m; *d* represents the distance between the signal transmitter and the signal receiver; *a* represents the channel attenuation index, in dB/m, and the typical apartment and office environment value is 0.2 m; *γ*_*SE*_ indicates the index value of the same building floor test. In different types of coverage areas, the value of *γ*_*SE*_ is different.

In the indoor environment, the attenuation factor model can be selected as the indoor wireless propagation model, and its expression is:

(2) $$\begin{array}{c} PL\left(d\right)\left[dB\right]=PL\left(d_{0}\right)+10n\mathrm{lg}\left(\frac{d}{d_{0}}\right)+FAF. \end{array}$$

The two-way relay transmission of the system is divided into two stages: multiple access stage (the first time slot) and transmission stage (the second time slot). In the multiaccess stage, all users send information to the relay station at the same time. In the transmission phase, the relay node amplifies the received information and sends it to the receiver. The two-way relay security network system model is shown in Figure 4.

Assume that each user group *k* is composed of *A*_*k*_, *B*_*k*_, and the bandwidth of each subchannel is *B*, and it is divided into *N* subchannels. Assume that in the multiple access stage, the user *A*_*k*_, *B*_*k*_ occupies the subchannel *i*, and the signal received by the relay node is

(3) $$\begin{array}{c} Y_{EN}^{i}=\sqrt{p_{A_{k}}^{i}g_{A_{k},RN}^{i}}X_{A_{k}}^{i}+\sqrt{p_{B_{k}}^{i}g_{B_{k},RN}^{i}}X_{B_{k}}^{i}+Z_{RN}^{i}, \end{array}$$

where *X*_*A*_*k*__^*i*^, *X*_*B*_*k*__^*i*^ are the transmission signal of *A*_*k*_, *B*_*k*_ on subchannel *i*, *p*_*A*_*k*__^*i*^, *p*_*B*_*k*__^*i*^ are the emission power of *A*_*k*_, *B*_*k*_, *g*_*A*_*k*_,*RN*_^*i*^, *g*_*B*_*k*_,*RN*_^*i*^, respectively, represents the channel gain from *A*_*k*_, *B*_*k*_ to relay station *R* on subchannel *i*, and *Z*_*RN*_^*i*^ is that the average value of relay node *RN* on subchannel *i* is 0.

In the broadcast stage, the signals received by *A*_*k*_, *B*_*k*_ and eavesdropper *E* on subchannel *j* are

(4) $$\begin{array}{c} Y_{A_{k,j}}^{j}=\xi \sqrt{p_{RN}^{j}}h_{A_{k}}^{j}Y_{RN}^{i}+Z_{A_{k}}^{j},\\ Y_{B_{k,j}}^{j}=\xi \sqrt{p_{RN}^{j}}h_{B_{k}}^{j}Y_{RN}^{i}+Z_{B_{k}}^{j},\\ Y_{E_{i}}^{j}=\xi \sqrt{p_{RN}^{j}}h_{E}^{j}Y_{RN}^{i}+Z_{E}^{j}, \end{array}$$

where *j* ∈ {1,2, ⋯, *N*} is the subchannel occupied by the relay node in the broadcast stage; *ξ* is the forwarding amplification factor of the relay node; *h*_*A*_*k*__^*j*^, *h*_*B*_*k*__^*j*^, *h*_*E*_^*j*^ are the channel gain of relay node *RN* to *A*_*k*_, *B*_*k*_, *E* on subchannel *j*, respectively; *p*_*RN*_^*j*^ is the transmitting power of the relay node on the subchannel *j* in the broadcast stage; and *Z*_*A*_*k*__^*j*^, *Z*_*B*_*k*__^*j*^, *Z*_*E*_^*j*^ are the white Gaussian noise of *A*_*k*_, *B*_*k*_, *E* on subchannel *j*, respectively.

Each vertex in the minimum rigid graph has at least two adjacent edges [17], so the minimum rigid graph has less communication complexity and stronger robustness. Especially, the singular value of the stiffness matrix provides a method to measure the algebraic properties of the network [18]. Define the stiffness matrix of edges in the network as follows:

(5) $$\begin{array}{c} X_{\left(G,P\right)}={\bar{M}}_{\left(G,P\right)}{\bar{M}}_{\left(G,P\right)}^{T}\in R^{\left|\varepsilon \right|\times \left|\varepsilon \right|}. \end{array}$$

Among them, rigid graphs with larger determinant eigenvalue have better algebraic stiffness characteristics. Good stiffness characteristics can ensure that the network coverage positioning has a small error, thus improving the stability of the network.

Under the condition that the graph is the minimum stiffness graph, the trace value of the stiffness matrix can be maximized. This process can be transformed into an optimization problem:

(6) $$\begin{array}{c} \underset{\varepsilon }{\text{maximize}}\text{ trace}\left({\bar{M}}_{G,P}{\bar{M}}_{G,P}^{T}\right),\\ \text{subject to rank}\left({\bar{M}}_{G,P}\right)=2n-3. \end{array}$$

This optimization problem can be solved by a classical greedy algorithm.

The coverage areas of base stations are not exactly the same. Therefore, a weight coefficient is introduced to correct it. This weight coefficient is determined by the ratio of user density to base station capacity. If the ratio is larger, the coverage radius will be smaller. On the contrary, it should be larger. Switching decision formula is

(7) $$\begin{array}{c} Mn+Ocn-Hys>Ms+Ocs+off, \end{array}$$

where *Mn* represents the measurement result of the neighboring cell, *Ocn* represents the specific offset of the neighboring cell, *Ms* represents the measurement result of the serving cell, *Ocs* represents the specific offset of the serving cell, *Hys* represents the delay of the event, and *off* is the offset value of the event [21].

## 4. Experiment and Results

### 4.1. System Test Analysis

System performance testing is an important task in the testing task. When designing performance test cases, this system adopts the method of continuous iterative improvement, that is, the iterative process of testing, improvement, and retest. At the same time, when testing the performance of the system, it is not entirely based on test cases, but the test plan is adjusted in time according to the actual situation to meet the needs of the test system. Independent business performance test is actually the concurrent performance test of a business of the core business module, which can be understood as a unit performance test. Composite business performance testing is the concurrent performance testing of multiple services from one or more modules. The stress test scenario of concurrent user access is shown in Figure 5.

It can be seen from Figure 5 that when the number of users is less than 800, the response time of the system increases steadily with a slope. When the number of users is close to 1,000, the system drops obviously, and the drop is very serious, and a red line warning appears. Therefore, when less than 800 users access the system, the system performance may be in a stable state. If there are more than 1,000 users, there is a problem with the system performance. Try to keep it below 800. For the test of the improved system, the users who participated in the test of the existing management system before are still invited. The relevant data of six users who completed the usability task are shown in Table 1.

After completing the task, each user needs to fill out the scale. The number 1 stands for “very different,” and 5 stands for “very much agree.” The scores of the six user scales calculated are shown in Table 2.

The test results show that the improved user satisfaction is 62.23, and the user satisfaction has been improved to some extent. When users view a page, they do not need to think or spend a little time thinking to understand what the content on the page means and how to act. There is still a lot of attribute information in the real talent data, which can be gradually added in future applications. Keeping the attributes that have a great influence on outstanding talents' achievements and removing the attributes that have little influence will make the model more scientific and complete, and the prediction results will be more accurate.

Therefore, curriculum development must be based on a complete workflow, in-depth analysis of the workflow, and flawless integration of the entire production industry. Courses from various disciplines, occupations, and degrees should all be taken into account when creating a curriculum structure. Basic professional knowledge, interdisciplinary knowledge, professional ability, comprehensive application ability, and comprehensive ability should all be covered in the curriculum. The human society in the AI era is a complex multiparty coordination system, with real-world and virtual-world governance coexisting. This necessitates a re-examination of stakeholder relationships and a re-definition of governance scope in vocational college education. Continuous innovation and progress are required to strengthen the synergy of various stakeholders and to realize the Pareto optimal governance mechanism of vocational college education, such as restraint, encouragement, and guarantee.

Therefore, the professional training system in the AI era should no longer be limited to providing procedural training content for the workforce, such as computer science, data analysis, and so on, but should provide people-to-people training, machine training, and communication skills training between people and the world; provide training to deal with sudden problems; and provide training in critical cognition and thinking and cognition. The provision of these training contents will surely pave the way for the smooth transition of the labor force to the AI era.

### 4.2. Analysis of Wireless Network Optimization Algorithm

In order to verify the accuracy of the algorithm, this section uses MATLAB software to conduct simulation experiments to verify the effectiveness of the algorithm. The algorithm in this document is compared with other different algorithms, and the number of user groups is 18. In all simulations, the flat fading channel gain can be modeled by a unit random variable, which follows the average exponential distribution, and the path loss index is set to 3.

Figure 6 counts the traces of the stiffness matrix of the topological graph generated from the algorithm of reference [18] based on the topology of the least rigid graph and the least rigid graph constructed by the algorithm in this paper.

It can be seen from Figure 6 that in the same environment, the minimum rigid graph constructed by the algorithm in this paper has a large trace, which indicates that the minimum rigid graph generated by the algorithm has a good algebraic performance of stiffness, which is conducive to enhancing the stability of the network.

Drop call rate is an important indicator in mobile communication, which refers to the probability of unexpected interruption of communication in the process of mobile communication. Drop call rate reflects the communication quality of mobile networks to some extent. To illustrate the problem here, eight communities are selected from five sites. These five selected sites are macrosites, which are scattered and basically scattered in the whole cluster area. Then compare the relationship between your deviation and network indicators to guide optimization and replacement. The deviation here includes the absolute error between the physical site and the logical site and its replacement error. Figures 7 and 8 show the relationship between the adjusted wireless network index and polygon deviation.

According to the experimental data, it can be seen that the overlapping coverage deviation is obvious. When the absolute deviation is greater than 2, the network index fluctuates obviously, and the overall trend is upward, which increases with the increase of deviation. In the process of constructing the minimum stiffness graph, the edges are sorted in ascending order at first, and then the edge with the largest trace of the stiffness matrix is selected to join the stiffness matrix, that is, the communication link weight of the edge is further reduced while ensuring the algebraic performance of network stiffness. In the simulation, it is assumed that there is a relay node, an illegal *E*, and multiple legitimate users on the network. Users are randomly distributed in a circle with a radius of 50 meters centered on the relay node (all users are within the coverage of the relay node). Here, it is assumed that the distance between *E* and the relay node varies between 100 and 400 meters, and the total transmission power of the relay is set to 1,000 mW as shown in Figure 9.

It can be seen that when *E* is far away from the relay node, the average satisfaction of the user group shows an upward trend. When *E* is far away from the relay node, the signal-to-noise ratio it receives decreases, and the more and less communication information *E* can steal, the higher the security satisfaction of users will be. When *E* leaves the relay node within 250 meters, the average security satisfaction of all user groups increases rapidly. It is also found that within the range of 250 m, the user security satisfaction of the optimized algorithm in this paper is 0.93, and the user security satisfaction of the proposed optimized algorithm is higher than that of other algorithms. As *E* is far away from the relay node, this gap will become smaller and smaller.

## 5. Conclusions

The rise of AI has created a new demand for talent, requiring vocational colleges to adjust and reshape talent development goals in response to changing industry structures. As a result, establishing an educational talent training system in vocational colleges that incorporates AI technology can help mitigate the impact of AI on vocational college employees. The project developed a design scheme for a vocational college education talent management system based on a wireless network after conducting extensive field research to meet the needs of enterprise talent management in the AI era. The system essentially performs the expected system design function, and it has undergone a series of system tests. The results of the tests show that the system is functional and robust. The talent management system's wireless network optimization results show that within a range of 250 m, the optimized algorithm in this paper's user security satisfaction is 0.93, and the satisfaction of the optimized algorithm proposed by user security is higher than that of other algorithms. It demonstrates that the algorithm has good algebraic connectivity and stiffness properties.

## Figures and Tables

**Figure 1:** Talent management platform.

**Figure 2:** System function module structure.

**Figure 3:** Overall structure diagram of data mining system.

**Figure 4:** Two-way relay security network system.

**Figure 5:** User concurrent access test.

**Figure 6:** Trace of the stiffness matrix.

**Figure 7:** Relationship between the absolute deviation of different stations and deviation of handover success rate.

**Figure 8:** The relationship between the absolute deviation of different stations and the deviation of dropped call rate.

**Figure 9:** The relationship between the distance from *E* relay and users' safety satisfaction.

**Table 1:** Completion rate and average time of tasks.

Task 1			Task 2		
Complete the task	After being prompted, the task is completed	Average completion time	Complete the task	After being prompted, the task is completed	Average completion time
100%	0	15 s	88.3%	9.6%	20 s

**Table 2:** User scale score.

User	Score
1	55
2	63
3	71
4	66
5	62.1
6	56.3

## Data Availability

The data used to support the findings of this study are available from the corresponding author upon request.

## References

[1] Huang Z., Liu Y., Zhan C., Lin C., Cai W., Chen Y. (2021). A novel group recommendation model with two-stage deep learning. *IEEE Transactions on Systems, Man, and Cybernetics: Systems*.

[2] Stukalina Y. (2010). The management of integrated educational environment resources: the factors to be considered. *European Journal of Education*.

[3] Ginsburg S., van der Vleuten C., Eva K. W., Lingard L. (2015). Hedging to save face: a linguistic analysis of written comments on in-training evaluation reports. *Advances in Health Sciences Education*.

[4] Leńko-Szymańska A. (2014). Is this enough? A qualitative evaluation of the effectiveness of a teacher-training course on the use of corpora in language education. *ReCALL*.

[5] Derosa N. M., Fisher W. W., Steege M. W. (2014). An evaluation of time in establishing operation on the effectiveness of functional communication training. *Journal of Applied Behavior Analysis*.

[6] Santos Filho S. B., Souza K. V. (2020). Metodologia para articular processos de formação-intervenção-avaliação na educação profissional em enfermagem. *Ciência & Saúde Coletiva*.

[7] Chen J., Du C., Zhang Y., Han P., Wei W. (2021). A clustering-based coverage path planning method for autonomous heterogeneous UAVs. *IEEE Transactions on Intelligent Transportation Systems*.

[8] Zhang J., Feng W., Yuan T., Wang J., Sangaiah A. K. (2022). SCSTCF: spatial-channel selection and temporal regularized correlation filters for visual tracking. *Applied Soft Computing*.

[9] Zheng K.-n., Sun S.-m., Yu H. (2016). College teaching quality evaluation based on system dynamics model. *MATEC Web of Conferences*.

[10] Sun M.-h., Li Y.-g., He B. (2017). Study on a quality evaluation method for college English classroom teaching. *Future Internet*.

[11] Chen Y. (2021). College English teaching quality evaluation system based on information fusion and optimized RBF neural network decision algorithm. *Journal of Sensors*.

[12] Dong Q. W., Wang S. M., Han F. J., Zhang R. D. (2019). Innovative research and practice of teachers’ teaching quality evaluation under the guidance of ‘innovation and entrepreneurship’. *Procedia Computer Science*.

[13] Yang X. (2017). Research on the teaching quality evaluation of law course in colleges based on the AHP model. *Revista de la Facultad de Ingenieria*.

[14] Liu W., Zhao S., Li X. (2014). The practice of advanced mathematics teaching quality evaluation system. *Proceedings of the 2012 International Conference on Cybernetics and Informatics*.

[15] Jian Q. (2019). Multimedia teaching quality evaluation system in colleges based on genetic algorithm and social computing approach. *IEEE Access*.

[16] Sagduyu Y. E., Shi Y., Fanous A., Li J. H. (2017). Wireless network inference and optimization: algorithm design and implementation. *IEEE Transactions on Mobile Computing*.

[17] Xiao F., Xie X., Li Z., Deng Q. A. L. (2018). Wireless network optimization via physical layer information for smart cities. *IEEE Network*.

[18] Zhang P., Ding X., Xu J., Wang J. L. (2020). Successive interference cancellation based throughput optimization for multi-hop wireless rechargeable sensor networks. *Sensors*.

[19] Wang R., He G., Wu X., Wang F., Hu Y. (2017). Multicast optimization and node fast location search method for wireless sensor networks based on ant colony algorithm. *Journal of Digital Information Management*.

[20] Wang S. (2021). Design of minimizing expected energy of multisource wireless cooperative network based on multiobjective optimization. *Mobile Information Systems*.

[21] Singh S., Mitra D., Baghel R. K. (2021). Wireless powered communication network optimization using PSO-CS algorithm. *Wireless Networks*.

[22] Daniel J., Francis S. F. V., Velliangiri S. (2021). Cluster head selection in wireless sensor network using tunicate swarm butterfly optimization algorithm. *Wireless Networks*.

[23] Kakadia D., Ramirez-Marquez D. J. E. (2020). Quantitative approaches for optimization of user experience based on network resilience for wireless service provider networks. *Reliability Engineering & System Safety*.

